The article "Short-Term Demand Forecast of E-Commerce Platform Based on ConvLSTM Network" was published in 2022. Journal: Comput Intell Neurosci.

# Short-Term Demand Forecast of E-Commerce Platform Based on ConvLSTM Network

**DOI:** 10.1155/2022/5227829

**Published:** 2022-07-14

**Authors:** Zan Li, Nairen Zhang

**Affiliations:** ^1^College of Business, Zhengzhou College of Finance and Economics, Zhengzhou 450000, China; ^2^Department of Decision Consultation, Henan Administration Institute, Zhengzhou 451000, China

## Abstract

Based on real sales data, this article constructed LGBM and LSTM sales prediction models to compare and verify the performance of the proposed models. In this article, we forecast the product sales of stores in the future *T* + 3 days and use MAPE as the evaluation index. The experiment shows that the product sales prediction model based on the convolutional LSTM (ConvLSTM) network has better prediction accuracy. From a store point of view, ConvLSTM prediction model MAPE was 0.42 lower than the long short-term memory (LSTM) network and 0.68 lower than LGBM. From the perspective of commodity categories, different commodity categories are suitable for different forecasting methods. Some categories are suitable for regression forecasting, while others are suitable for time-series forecasting. Among the categories suitable for time-series forecasting, the ConvLSTM model performs the best.

## 1. Research Background

In recent years, the Internet has developed rapidly with the passage of time, and enterprises have accumulated massive valuable data, which contains a huge value and is waiting for people to dig. In addition, due to the rise of big data and artificial intelligence, our life has undergone great changes, and many emerging fields of science and technology have emerged. Traditional enterprises also want to take the ride of big data and artificial intelligence to bring scientific analysis and guidance to companies and enterprises.

New retail, supported by artificial intelligence, big data, mobile Internet, and other cutting-edge technologies, emerges in the trend of China's residents' consumption upgrading. With new concepts such as scenarioization, fragmentation, and experientialization, new retail formats are reconstructed, leading to the transformation and upgrading of China's retail market. The traditional retail has come to the stage of contraction, the development of traditional e-commerce has reached a bottleneck today, and the sales industry is in a very challenging period. In the near future, the traditional offline or pure online form may no longer exist, and the full integration of online and offline new retail will be the general trend.

While the new retail industry has been changed, there are also many new challenges. Competitors from a variety of online and offline channels and an increasingly rich variety of goods, especially in the face of changing user needs, force enterprises to constantly make adjustments in the process of pursuing market profits [1]. The development direction of new retail is still to meet the changes of users' needs. As a result, predicting users' needs accurately is very important and presents more challenges in the context of the new retail industry.

The article "Short-Term Demand Forecast of E-Commerce Platform Based on ConvLSTM Network" was published in 2022. Journal: Comput Intell Neurosci.

## 2. Related Works of Demand Forecasting

Research on demand forecasting has always been a hot topic for experts at home and abroad. Accurate forecast results are extremely important in different industries, especially for the emerging new retail, which will directly affect the sales of enterprises. Combined with the research of domestic and foreign experts on demand forecasting, the forecasting method is divided into qualitative forecasting and quantitative forecasting.

Qualitative sales forecasting methods mainly include the subjective probability method, expert judgment opinion method, Delphi method, mutual influence method, scenario prediction method, etc [2–4]. Quantitative sales forecasting methods mainly include the time-series method (e.g., autoregressive series analysis [5], ARIMA model [6]), machine learning method [7] (e.g., artificial neural network [8, 9], extreme learning machine [10], support vector machine (SVR) [11], and ensemble algorithms), and deep learning method.

Because the qualitative prediction method is mainly to predict the future demand through experts combined with their rich business experience, this method is more applicable when there are few influencing factors and the sales information cannot be fully quantified. However, due to its shortcomings such as subjective factors and poor reproducibility, in the face of an increasingly complex business environment, this method is not accurate in demand forecasting. Therefore, this article mainly expounds the research status of demand forecasting at home and abroad from the quantitative forecasting methods, namely the time-series method, machine learning method, and deep learning method.

### 2.1. Time-Series Prediction

Autoregressive series analysis is one of the most popular methods in time-series application, which only uses single-dimension sales data for forecasting. Back in 1927, some mathematicians proposed the earliest autoregressive model for analyzing sequence data, referred to as the AR model [12]. On the basis of the AR model, scientists combined the autoregressive process AR with the moving average process MA to produce the autoregressive moving average model, referred to as ARMA [13, 14]. AR and ARMA models have good model effects when facing stationary time-series scenes, but they are not suitable for nonstationary sequence scenes which are common. Therefore, people consider introducing difference transformation to stabilize them and generate the differential autoregressive moving average model with difference transformation, ARIMA for short [15].

The article "Short-Term Demand Forecast of E-Commerce Platform Based on ConvLSTM Network" was published in 2022. Journal: Comput Intell Neurosci.

For example, researchers used the beverage sales data of an enterprise, which only included sales data without other additional features; established stationary series models such as MA and ARMA for analysis and prediction, respectively, and nonstationary ARIMA models for comparative analysis; and obtained very ideal prediction results. In 2018, Facebook opened the time-series prediction algorithm Prophet, which represents the time series as the sum of trend term, period term, holiday term, and error term, which can well fit and predict the time series in the business field.

### 2.2. Machine Learning Prediction

With the development of machine learning, it is found that the time-series problem can be transformed into a machine learning regression problem, that is the future target data can be regression as “label.” This method can not only use the sales dimension, but also add time, holidays, weather, and other characteristics of different dimensions. Common machine learning algorithms include support vector regression (SVR) algorithm, decision tree regression algorithm, Leo Breiman and Adele Cutler-proposed bagging ensemble learning on the basis of decision tree, and the random forest algorithm generated by the fusion of multiple decision trees. Boosting ensemble learning is introduced, which iterates multiple base learning devices, and the generated GBDT algorithm, a series of extended tree model algorithm, and an artificial neural network can solve the regression problem [16].

Avanija et al. used XGBoost to predict the house price in 2021 [17], which improved the accuracy of sales forecast and realized effective control of inventory. Experimental results show that XGBoost can fully consider the influence of external factors and historical data on sales volume and effectively predict sales volume. SVR model is used to predict the sales volume [18]. Through comparative experimental analysis with the ARIMA model and linear regression model, it was proved that the SVR model has higher prediction accuracy. Because the SVR algorithm can transform complex nonlinear regression problem into linear regression problem of high-dimensional feature space, it can be widely used in various time-series prediction problems, such as weather prediction, traffic flow prediction, etc.

### 2.3. Deep Learning Prediction

In recent years, with the growing enterprises accumulating the amount of data, the sales environment is becoming more and more complex and the traditional prediction method of machine learning also exposed the shortcomings, such as training time being too long, it is not easy to convergence. Therefore, people have thought more deeply about the prediction model and started to use deep learning methods to build the prediction model [19]. In terms of prediction, Shih et al. proposed a model to forecast short-term goods demand in an e-commerce context [20]. They found that short-term demand for goods could not be predicted by the periodicity of historical data, so they built a database based on buyers' reviews to predict short-term demand for goods from this unique perspective. Based on the combination of traditional statistical model and deep learning model, the demand for e-commerce products is predicted, and good prediction results are obtained [21].

The article "Short-Term Demand Forecast of E-Commerce Platform Based on ConvLSTM Network" was published in 2022. Journal: Comput Intell Neurosci.

## 3. Sales Forecasting Modeling

The sales volume forecast of commodities can be predicted by the regression method, or the sales data can be fitted by time series. Whether regression prediction or time-series prediction, there is a specific assumption that the features are independent of each other, and the samples are independent of each other. Features are independent of each other and can be solved by constructing associative features. However, the samples are independent of each other, and there are some defects in the scenario where multiple commodities need to be predicted, that is the interaction between different commodities is not considered. There is a certain relationship between commodities, which are mutually exclusive and complementary. Some commodities are of the same type. If you select commodity A, you will not select commodity B with the same attributes. Similarly, some commodities have complementary relationships and can be sold together, after you select commodity A, you need to match commodity C.

This chapter introduces the sales prediction model based on related commodities. Word2Vec model is used to group the predicted commodities first, and then the ConvLSTM network is used to predict the sales of the commodities after grouping in the future *T* + 3 days, as shown in Figure 1. First, Word2Vec is used for low-dimensional spatial mapping of feature words, which can make words with similar context have similar spatial mapping and extract the semantic characteristics of words. Starting from the receipt data of goods, the vector representation of goods is obtained, so as to extract the association of different goods. Then, ConvLSTM can learn the long-term dependence of data and extract the spatial characteristics of data to predict the sales volume of associated goods.

The article "Short-Term Demand Forecast of E-Commerce Platform Based on ConvLSTM Network" was published in 2022. Journal: Comput Intell Neurosci.

### 3.1. Commodity Association Clustering Based on Word2Vec

At present, there are many association analysis algorithms, such as Apriori and FP-growth. The basic idea is to select the commodity combination with high frequency by counting various commodity combinations. However, these algorithms have some disadvantages, they need to traverse all the collections in the data set globally, which consumes a lot of time. At the same time, in the face of a large amount of data, the commodity associations that can be mined are limited.

Word2Vec is a shallow neural network model, which is often used for natural language tasks. It can map feature words into low-dimensional word vectors and map semantically similar feature words into similar projection spaces. First, we need to build a Word2Vec model for commodity ticket data, train the vector representation of commodities, and then conduct association clustering according to the vector representation of commodities.

#### 3.1.1. Commodity Word Vector Model

The vector representation of Word2Vec training commodity needs to be preprocessed for commodity receipt data according to the input requirements of the model, and then appropriate training methods are selected for unsupervised learning. Finally, the vector mapping space of the commodity is obtained. In the model, the vector space of the commodity is the network parameters from the input layer to the hidden layer.

*(1) Data Preprocessing*. To train the word vector of goods by using the receipt data of goods, the receipt data need to be processed according to the algorithm requirements of the Word2Vec model. The discovery of receipt data shows that (1) there are some dirty data in receipt data, such as shopping bags, price difference compensation, and returns; (2) the same user makes multiple receipts when shopping at one time; (3) the user buys fewer goods; and (4) there are multiple same goods in the same receipt.  Figure 2 shows the processing process of receipt data.

First, it is necessary to remove the dirty data in the data and delete nonpredictive goods in the receipt. These dirty data are similar to stop words in natural language, which will interfere with model training and destroy the mapping space of vectors. Then, data integration is carried out on the receipt data. There may be multiple receipts for one user and multiple same goods in one receipt. We need to summarize the goods purchased by the same user in the same day and then eliminate the duplicate goods in the receipt data.

Word2Vec model is a three-layer neural network, which predicts its context according to known characteristics or predicts the feature word according to the context of the feature word. The input of the model is the unique heat coding of the known feature word. When used for vector representation of goods, it is necessary to carry out unique thermal coding for the goods contained in the invoice data first and establish a mapping dictionary to transform the goods into the form of unique thermal coding before the commodity input model is known.

*(2) Commodity Word Vector Training*. Word2Vec has two models. CBOW model is used this time. The input layer is other commodities in the same receipt data of the commodity to be predicted, and the output layer is the one-hot vector of the predicted commodity.

The article "Short-Term Demand Forecast of E-Commerce Platform Based on ConvLSTM Network" was published in 2022. Journal: Comput Intell Neurosci.

When training the Word2Vec model, you need to set the size of the context window, and the dimension of the word vector. In general, the input is 2*n* commodities up and down the commodity *w*_*t*_, because the location relationship of commodities is not considered in the receipt data, the user checks out randomly during shopping, and any commodity in the ticket data should be associated with other commodities in the same ticket. Therefore, *n* should include all commodities as much as possible. Assuming that the total number of commodities in the ticket is *m* at most, *n*=*m* − 1 should be set.

As for the dimension of the word vector, the decisive factor is the number of neurons in the hidden layer *N*, and the input data are spatially mapped through matrix *W*_*V*×*N*_, where vector {*h*_1_, *h*_2_,…, *h*_*i*_,…, *h*_*n*_} is the commodity of commodity *w*_*t*_ and *W*_*V*×*N*_ is the transfer matrix of the transformation of the word vector.

#### 3.1.2. Commodity Association Clustering

According to the commodity vector trained by Word2Vec, the commodities are correlated and clustered. Similar commodities have similar distances. The clustering algorithm can be used to group commodities and predict the relevance of commodities. The commonly used clustering algorithms include K-means clustering, mean-shift clustering, DBSCAN clustering, expectation-maximization (EM) clustering using Gaussian mixture Model (GMM) clustering, hierarchical clustering, etc. Each clustering has its advantages and disadvantages, and it is necessary to select the appropriate clustering method according to the manifestation of data samples.

In combination with the vector representation of commodities, this article will select the appropriate clustering method based on K-means clustering and DBSCAN clustering. K-means clustering is a clustering algorithm based on partition. Its main idea is to make the spacing of data samples within clusters as small as possible and the spacing of samples between clusters as large as possible, and it is a local optimal algorithm, and the results of multiple clustering will be different. The time complexity of the K-means algorithm is low, and the algorithm has excellent performance and high efficiency when facing the scene of large data sets. However, the algorithm is sensitive to outliers, and the selection of the total number of cluster classes and the initial cluster center has a great influence on the clustering effect. K-means is suitable for processing data sets with spherical data distribution.

The article "Short-Term Demand Forecast of E-Commerce Platform Based on ConvLSTM Network" was published in 2022. Journal: Comput Intell Neurosci.

Among the clustering algorithms, DBSCAN clustering is based on density, the general idea is to find a high density of samples first. Then the high density around samples will gradually come together, eventually forming a cluster around each sample point. However, unlike K-means clustering, DBSCAN does not specify the number of clusters to be formed. Under the same settings, the results of multiple DBSCAN clustering are consistent. The advantage of DBSCAN is that it is insensitive to noise and can cluster clusters of different sizes and arbitrary shapes. However, it is sensitive to the radius of the circle and the threshold value of samples in the circle. When the density of data clusters is different, it is difficult to select an appropriate radius, thus affecting the clustering effect. DBSCAN works with clusters of any shape, but requires roughly the same density between clusters.

Through data visualization, it can be found that the total number of commodities to be clustered is not large, which is 500, the distribution of commodity vectors is irregular, there is a small amount of noise, and the density between clusters is roughly the same. Therefore, the DBSCAN algorithm is selected to represent the association clustering of commodity vectors. Taking the vector representation of 500 commodities trained by Word2Vec as input, using the DBSCAN algorithm, the distance threshold EPS is set as 0.1 and the sample number threshold min_Samples as 10, and the Euclidean distance is used as the distance measurement parameter to cluster the commodities.

## 4. Forecast Model of Commodity Sales Based on ConvLSTM

In the previous chapter, we constructed a commodity relevance clustering model based on Word2Vec, whose practical significance is to mine the association relationships between different products, the input of ConvLSTM prediction model is constructed, and the prior knowledge of product association is integrated. This section will mainly introduce the commodity sales forecast model based on ConvLSTM, including model input and output, network structure design, activation function selection, model training, etc.

The article "Short-Term Demand Forecast of E-Commerce Platform Based on ConvLSTM Network" was published in 2022. Journal: Comput Intell Neurosci.

### 4.1. Input and Output Structure Design of Network

The product sales forecast based on ConvLSTM is actually a supervised learning, which uses the sales data of stores to predict the product sales on the *n*th day in the future. Input data should not only contain sales data, discount information, and time characteristics of stores, but also conform to the requirements of the ConvLSTM neural network for input data.

In the figure, we splice the data of *N* days before time *T* into a two-dimensional tensor, and then sort these two-dimensional tensors according to time, thus forming an example of neural network input. It is worth noting that each two-dimensional tensor is combined according to the sales situation of each commodity and the results of commodity association clustering. Among them, the two-dimensional tensor acts as the time-sharing sales volume of a single commodity in each time period every day, and the column first puts the similar commodities in each cluster together according to the clustering results of commodities, and then according to the distance between clusters, the clusters close to each other are combined to arrange all the commodities to be predicted.

*S*_*T*_ can be considered as the sales data of the day *T*, then each example is composed of samples {*S*_*T*−*H*_,…, *S*_*T*−*I*_,…, *S*_*T*−1_, *S*_*T*_} and lable, where *H* is the number of ConvLSTM network neurons, that is the sales data of consecutive *H* days in history input at one time, *N* is the time span to be predicted, and the output of ConvLSTM network is the sales data *S*_*T*+*N*_ of the *T* + *N* day. The input of the whole model requires *S*_*T*_ fusion with other external data of the day *T*, which will be explained in detail in the model network design in the next section.

### 4.2. Model Network Design

LSTM network model is very suitable for dealing with problems with time-series characteristics. The network transmits information according to the forward propagation of time step, and the cell state will be updated gradually, and the information is transmitted and forgotten through three gated systems. LSTM sales prediction model can add a feature extraction layer before data input LSTM to improve the prediction effect. For example, the prediction model based on the WaveNet-LSTM network adds a layer of the WaveNet network before the LSTM layer and uses causal convolution to obtain local and global information of the whole time series.

The convolutional neural network has a strong representation learning ability and can recognize features of different locations in space by using convolution operation and pooling operation of data samples. The convolutional neural network takes advantage of the feature that convolution operation can capture local information of data and uses multiple filters (convolution kernel) to extract information at the same time, thus realizing local perception to obtain global information. In this chapter, the advantages of convolution operation for spatial feature extraction will be utilized, and the vector operation of LSTM will be replaced by convolution operation, and combined with external influencing factors of sales volume, a sales prediction model for associated goods will be constructed. The model network diagram is shown in Figure 2.

The article "Short-Term Demand Forecast of E-Commerce Platform Based on ConvLSTM Network" was published in 2022. Journal: Comput Intell Neurosci.

The model is divided into two parts. In the first part, the store's sales characteristics, discount information, time characteristics, and other features are fused to form the input of the ConvLSTM network. For the input data of the model, first, the attribute features such as daily discount information and time features are fully connected, then the extracted feature reshape is the same size as the sales feature, and finally the concat operation is used to form the input of the ConvLSTM network for the sales features and the reshaped features. The second part consists of a ConvLSTM network prediction module, which consists of a ConvLSTM network layer and a fully connected layer. After the extracted features are inputted into the network, the prediction information is outputted, and the final prediction result is obtained through the full connection layer.

ConvLSTM network can be used to extract time-series characteristics and spatial characteristics of sales volume of various commodities for the following reasons:

First, traditional sales forecasting methods assume that different commodities are independent of each other and can only forecast independent commodities. The prediction method based on time series can use single-dimension sales data to forecast, but only one kind of commodity can be predicted. To forecast multiple commodities, multiple models need to be constructed. Regression-based prediction method can predict multiple commodities simultaneously by constructing feature engineering, but it cannot obtain time-series characteristics. The idea of the ConvLSTM network is to extract and transfer information of time series from two-dimensional matrix data, so that time-series prediction of multiple commodities can be made simultaneously.

Second, in real life, commodities often interact with each other. When shopping, people will consider the repetition and collocation of commodities. For commodities with repetitive functions, they will choose only one of them, while for commodities with complementary functions, they will buy them with each other. Based on this, the ConvLSTM network can not only capture the time-series characteristics of various commodities, but also extract spatial information of data and capture the interaction between commodities through convolution operation. However, the introduction of convolution operation may bring a series of problems, such as the selection of convolution kernel and poor fitting effect.

The article "Short-Term Demand Forecast of E-Commerce Platform Based on ConvLSTM Network" was published in 2022. Journal: Comput Intell Neurosci.

The model needs to capture the interaction between goods through the convolution operation, but convolution can only capture part of the local information; it is difficult to obtain global information, that is when there are too many goods, the convolution operation often cannot capture the association between goods with a long distance. If the convolution is extended, more commodity association information can be obtained at the same time, but too many parameters will affect the fitting effect. We integrate the association information of commodities in advance to obtain the prior knowledge of the association relations of commodities and put the commodities with certain association relations together, and then spliced them into the two-dimensional matrix form required by the network, so that even if the size of the convolution kernel cannot contain all commodities and cannot capture the association relation of commodities with relatively distant positions, the influence will not be great. In the process of data preparation, the relationship between goods located far away from each other is poor.

### 4.3. Selection of Activation Function

The activation function can introduce nonlinearity into the network model and enhance the expression ability of the model. In the gated mechanism of ConvLSTM, information is also forgotten and transmitted through activation functions, commonly used activation functions are as follows:

(1)   *The Sigmoid Function.* The sigmoid function expression is as follows:
  (1) $$\begin{array}{c} y=\frac{1}{1+e^{-x}}. \end{array}$$
Sigmoid is a commonly used nonlinear activation function. The value range of expression is [0, 1], and the range of derivative is [0, 0.25]. The function is easy to fall into the saturation zone on both sides, and the gradient disappears, and the output is not zero mean, which makes the model convergence slow.
(2)   *Tanh Function.* Tanh function is expressed as follows:
  (2) $$\begin{array}{c} y=\frac{e^{x}-e^{-x}}{e^{x}+e^{-x}}. \end{array}$$
The range of the Tanh function is [−1, 1], and the range of its derivative is [0, 1], which solves the problem that the sigmoid output is not zero mean value, but the problem of gradient disappearance still exists.
(3) *The ReLU Function.* ReLU function is expressed as follows:
  (3) $$\begin{array}{c} y=\max\left(0,x\right). \end{array}$$
When the input value of the function is greater than 0, the output of the ReLU function is equal to the input value. When the input value of the function is less than 0, the output is 0. Function can solve the problem of gradient disappearance in the process of model back propagation, but it can only be used in the hidden layer.

According to the network structure of ConvLSTM, the default activation function of input gate and output gate is the Tanh function, and its output range is [−1, 1]. However, according to the actual data, it can be found that most of the sales data of commodities are too large, which will change the distribution of data, cause the gradient to disappear, and the dimensions between different commodities are the same. If the data are forcibly normalized, some data will be extremely small, which will affect the effect of the model. In addition, when the sales data of commodities is relatively large, it is not necessary to consider the negative semi-axis when selecting the activation function. Therefore, the ReLU function is chosen.

The article "Short-Term Demand Forecast of E-Commerce Platform Based on ConvLSTM Network" was published in 2022. Journal: Comput Intell Neurosci.

### 4.4. Model Training

The training process of a neural network mainly includes two stages: the first stage is the forward propagation stage, and the second stage is the back propagation stage. Specifically, once the data set is ready and the model is built, model training can be carried out. First, it is necessary to set initial values for network parameters and then input model training data. Data samples enter the model network one by one and generate model predicted values through the forward propagation of network. The back propagation process uses an optimizer to update network parameters according to the error between the predicted value and the target value of the model until the termination condition of the model is met.

The effect of model training is affected by many factors, including initialization of parameters, selection of optimizer, selection of learning rate, etc.

#### 4.4.1. Initialization of Parameters

The training effect of the neural network model mainly depends on the updating of parameters by the optimizer. The optimizer back propagates the parameters through the gradient descent method, and the initialization of parameters greatly affects the convergence result of the model. If the initial value of the parameter is set too large, the gradient value of the parameter during back propagation will be too large, the gradient explosion will occur, and the amplitude of network update will be too large, which will make the model difficult to converge. If the initial value of the parameter is set too small, the gradient will be too small and the gradient will disappear, which will slow down the convergence speed of the parameter and make the model converge to the local optimal solution.

The article "Short-Term Demand Forecast of E-Commerce Platform Based on ConvLSTM Network" was published in 2022. Journal: Comput Intell Neurosci.

The initial value of network parameters should not be too large or too small and should keep the parameter positive or negative half as much as possible, and the expectation is 0. Network parameters can be initialized to small random numbers, such as random sampling with a Gaussian distribution with a standard deviation of 1 and mean of 0, or initialization with Xavier, but requires the activation function to be symmetric with respect to 0.

#### 4.4.2. Selection of Optimizer

In a neural network, parameter optimization mainly relies on the back propagation of the optimizer. The optimizer takes advantage of network errors, calculates gradients, and updates parameters so that the model approaches or achieves the optimal solution, that is, minimizes the objective function. The most basic optimizer is gradient descent, but in the optimization process, each epoch needs to consider all samples, which wastes time and occupies memory. In order to solve the inefficiency of the gradient descent method and accelerate the convergence speed, SGD (stochastic gradient descent) is introduced. Each iteration only uses one sample of all data to update the parameter gradient. Although SGD accelerates the model training speed, it will lead to convergence oscillation and lower accuracy, so it is not a globally optimal optimization algorithm. In order to accelerate the convergence of the model and improve the fitting accuracy, researchers also put forward a momentum optimization algorithm and adaptive learning rate optimization algorithm.

In this application, there is a large amount of actual data. A store has more than 300 examples a year, a total of more than 1000 stores, and the sales data will continue to increase and accumulate, and the data are sparse, so the Adam algorithm is selected. The Adam algorithm can adaptively change the learning rate of each parameter. It is very suitable for processing sparse data. It is not only conducive to the first-order distance estimation mean, but also makes full use of the gradient second-order distance estimation variance.

#### 4.4.3. Selection of Learning Rate

Learning rate is an important super parameter in network training; it plays a decisive factor in whether the objective function can converge to the local optimal value and how long it takes to converge to the optimal value. If the learning rate is small, the convergence speed of the model will become very slow. A small learning rate can ensure that the model will not miss any local optimal solution, but it will consume more time to make the model converge, especially when the model converges to the plateau area. When the learning rate is large, the model training speed becomes faster, but it may not converge, it is easy to cross the optimal value, and the gradient fluctuates back and forth around the optimal value.

The article "Short-Term Demand Forecast of E-Commerce Platform Based on ConvLSTM Network" was published in 2022. Journal: Comput Intell Neurosci.

Choosing an appropriate learning rate can ensure that the model can converge to the local optimal solution in a short time. This article will choose the method of learning rate attenuation to continuously adjust the learning rate in the training process. In the training process, a smaller learning rate training model is selected first and the learning rate after each round of iteration is gradually increased. By drawing a two-dimensional chart of learning rate and loss, we can find the optimal learning rate before the loss is no longer reduced.

## 5. Data Processing

### 5.1. Data Introduction

The data set of this experiment selects real commodity sales data of Q company, including sales statistics and receipt data of stores, covering four categories of commodities: meat, vegetables, cooked food, and aquatic products. This experiment selects the sales data of 5 stores, covering the period from January 1, 2017 to December 31, 2018, with a total of 11,393,481 pieces of data, including about 500 kinds of goods that appeared in the last 4 months.

### 5.2. Dividing Data Sets

In the experiment, the sliding window method is used to divide the data set, and the time step is 1 and the sequence length is 30. As shown in Figure 3, the feature in each example is the historical sales data of the store within 30 days, and lable is *T* + 3 to predict the sales volume of goods on the day.

## 6. Ablation Experiments

### 6.1. Comparison Method

The previous chapter mainly introduces the sales forecasting model based on the ConvLSTM network. This section will introduce the experimental comparison model, LightGBM prediction model, and LSTM prediction model. The two models will transform the sales forecasting model into a regression problem and a time-series problem, respectively:

1. LightGBM prediction model: GBDT is used as the base learner to make regression prediction of sales volume through feature engineering.
2. LSTM prediction model: it consists of one dense layer and one LSTM layer and then outputs the prediction results of the model through the full connection layer.

### 6.2. Parameter Setting

In experiment 1, the LightGBM prediction model, the features used are as follows: historical seven-day sales feature, time-sharing sales feature, pedestrian flow feature, weather feature, monthly feature, weekly feature, weekend feature, price change feature, promotion feature, temperature feature, weekly feature, and quarterly feature. The LightGBM prediction model adopts the grid search method for parameter tuning, and parameter settings are shown in Table 1.

The article "Short-Term Demand Forecast of E-Commerce Platform Based on ConvLSTM Network" was published in 2022. Journal: Comput Intell Neurosci.

In experiment 2, LSTM prediction model, the input data were first extracted through a Dense Layer to reduce the network parameters of the LSTM layer. Here, the dimension of the full connection layer was set as 1 ∗ 10, and the specific parameters of the model were set as follows:

1. *Optimizer*. Adam optimizer is selected to adaptively adjust the learning rate.
2. *Learning Rate.* Set this parameter to 0.001 in the experiment.
3. *Activation Function*. The three gating devices for information transmission in LSTM are equipped with activation functions, and the activation function is the ReLU function.
4. *Dropout Random Inactivation Rate*. To prevent overfitting, set dropout to 0.1.
5. *Error Function*. The error function is set as MSE in the experiment.
6. *Batch Size*. Batch size (batch_size) is set to 256 in the experiment.
7. *Iteration Times*. The training iteration times epoch is set to 1000 in the experiment.

Experiment 3 was based on the sales prediction model of the ConvLSTM network. In order to compare with experiment 2, the training mode of the ConvLSTM prediction model was the same as experiment 2. Adam optimizer was selected, and the learning rate was 0.001, etc. The difference is that ConvLSTM network will conduct convolution operation in the process of state transfer, and convolution-related parameters need to be set:

1. *Number of Convolution Kernels*. Here, the convolution kernels extract spatial features of two-dimensional data and set filters to 16.
2. *The Size of the Convolution Kernel*. In the experiment, the kernel_size of the convolution kernel is set to 10 ∗ 10.
3. *Convolution Step*. Set strides to (1,1).
4. *Zero-Complement Strategy.* In order to retain the convolution result at the boundary, the padding is set to the same in the experiment.

In this experiment, all models will be compared on the basis of the same original data set, and the model will predict the product sales within 3 days (*T* + 3) of the input data, and MAPE will be selected as the evaluation index of the model.

## 7. Analysis of Experimental Results

In this section, the prediction results of the three models will be compared and analyzed from two perspectives: the prediction results of the three models in different stores and the prediction results of the three models for different categories of goods. The prediction results used for comparison are all the best prediction results after the adjustment of the three models.

The article "Short-Term Demand Forecast of E-Commerce Platform Based on ConvLSTM Network" was published in 2022. Journal: Comput Intell Neurosci.

### 7.1. Comparison of Forecast Results of Different Stores

The comparison of the prediction errors of the three models in different stores is shown in Table 2, which shows the optimal performance of the three models in the evaluation index MAPE after the adjustment. On the whole, it can be seen that the prediction effect of the LSTM model is better than that of LGBM model. The average MAPE of the LGBM model's five stores is 38.98, which is 0.26 percentage points higher than that of the LSTM model. It can be seen that LSTM has advantages in dealing with time series, and the same applies when forecasting sales.

Most importantly, the ConvLSTM model performed best among the three prediction models, with an average MAPE of 38.3, 0.68 percentage points lower than that of the LGBM model and 0.42 percentage points lower than that of the LSTM model, indicating a significant performance improvement.

### 7.2. Comparison of Forecast Results of Different Categories of Commodities

As can be seen from the clustering results in the previous section, the whole commodity is divided into ten categories, six of which are selected in the experiment to show the prediction performance of the model in different categories, as shown in Table 3, and the comparison of prediction errors of the three models in different categories of commodity.

As shown in Table 3, the error performance of the three models is compared for different categories of goods. It can be found that models have different performance for different categories. For example, the LGBM model has better prediction effect for categories numbered 10001 and 10003, while the LSTM model and ConvLSTM model have better prediction effect for categories numbered 10002, 10004, 10005, and 10006. And the difference between the models is obvious. Categories 10001 and 10003 were suitable for regression prediction, and categories 10002, 10004, 10005, and 10006 were suitable for time-series prediction, and ConvLSTM outperformed LSTM in terms of the categories suitable for time-series prediction.

The above experiments show that the ConvLSTM model has better predictive performance than the LSTM model and LGBM model on the whole, but for individual commodities, some commodities are more suitable for regression prediction, and the LGBM model performs better. ConvLSTM network can learn the association information between goods through convolution operation and extract the dependence information of time series by LSTM, which realizes the capture of spatial information and time information and greatly improves the prediction ability of the model.

## 8. Conclusion

This article combines the real sales data set of Q company to make an example application of commodity sales forecasting model based on ConvLSTM. Before modeling, the data set was fully explored, and the whole modeling process of data preprocessing, feature engineering, and experimental result analysis was described in detail, in which the experimental result analysis made a detailed analysis of commodity clustering results, experimental comparison results, and model prediction effect. We found that by using ConvLSTM network, the model can not only extract the characteristics of time series, but also capture the characteristics of data space and predict the future sales of associated goods, and the ConvLSTM network model performs well in most of the time, but sales forecasting is a very complicated task, which is affected by many factors and still faces great challenges.

The article "Short-Term Demand Forecast of E-Commerce Platform Based on ConvLSTM Network" was published in 2022. Journal: Comput Intell Neurosci.

## Figures and Tables

**Figure 1:** The structure of the model.

**Figure 2:** Model network structure.

**Figure 3:** Data set partitioning by sliding window method.

**Table 1:** Parameter configuration of LightGBM sales prediction model.

Parameter	Setting
boosting_type	GBDT
objective	Regression
metric	MSE
nthread	5
learning_rate	0.01
num_leaves	25
max_depth	15
max_bin	255
subexample	0.8
co1example_bytree	0.8
feature_fraction	0.9
lambda_ll	0.1
lambda_12	0.0

**Table 2:** Comparison of forecast results of different stores.

Shop_Number	MAPE_LGBM	MAPE_LSTM	MAPE_ConvLSTM	MAPE_SVR	MAPE_ARIMA
101015	37.00	36.45	36.25	36.01	35.23
101016	40.31	39.83	38.50	37.1	38.21
101031	35.70	36.34	36.80	35.33	36.41
101044	40.83	41.95	40.00	39.89	38.98
101166	41.06	39.07	39.95	38.34	38.9
Mean value	40.98	38.728	38.03	37.34	37.55

**Table 3:** Comparison of prediction results for different categories.

Category_Number	MAPE_LGBM	MAPE_LSTM	MAPE_ConvLSTM	MAPE_SVR	MAPE_ARIMA
10001	36.65	39.72	42.86	35.45	36.67
10002	40.41	39.56	37.69	38.55	36.43
10003	38.50	41.88	41.32	39.41	37.54
10004	39.60	37.47	35.89	39.31	36.52
10005	40.46	41.04	39.52	38.99	38.12
10006	38.28	32.15	32.50	36.81	33.23
Mean value	38.92	38.64	38.02	38.08	36.41

## Data Availability

The experimental data used to support the findings of this study are available from the corresponding author upon request.
